The article "Prediction Models for One-Year Survival of Adult Patients with Acute Kidney Injury: A Longitudinal Study Based on the Data from the Medical Information Mart for Intensive Care III Database" was retracted in 2023. Reasons: suspected computer-generated content; unreliable results or conclusions; lack of ethics approval or compliance; missing or withdrawn patient consent.

# Prediction Models for One-Year Survival of Adult Patients with Acute Kidney Injury: A Longitudinal Study Based on the Data from the Medical Information Mart for Intensive Care III Database

**DOI:** 10.1155/2022/5902907

**Published:** 2022-07-05

**Authors:** Lifang Zhou, Laping Chu, Junqiong Peng, Shenhan Yin, Yafen Yu

**Affiliations:** Department of Nephrology, The Affiliated Hospital of Jiangnan University, Wuxi, Jiangsu 214000, China

## Abstract

Acute kidney injury (AKI) is a common complication of acute illnesses with unfavorable outcomes. This cohort study aimed at constructing prediction models for one-year survival in adult AKI patients based on prognostic nutritional index (PNI), platelet-to-lymphocyte ratio (PLR), neutrophil percentage-to-albumin ratio (NPAR), or neutrophil-to-lymphocyte ratio (NLR), respectively. In total, 6050 patients from Medical Information Mart for Intensive Care III (MIMIC-III) were involved. The least absolute shrinkage and selection operator (LASSO) regression was utilized to screen possible covariates. The samples were randomly divided into the training set and the testing set at a ratio of 7.5 : 2.5, and the prediction models were constructed in the training set by random forest. The prediction values of the models were measured via sensitivity, specificity, negative prediction value (NPV), positive prediction value (PPV), area under the curve (AUC), and accuracy. We found that NLR (OR = 1.261, 95% CI: 1.145–1.388), PLR (OR = 1.295, 95% CI: 1.152–1.445), and NPAR (OR = 1.476, 95% CI: 1.261–1.726) were associated with an increased risk, while PNI (OR = 0.035, 95% CI: 0.020–0.059) was associated with a decreased risk of one-year mortality in AKI patients. The AUC was 0.964 (95% CI: 0.959–0.969) in the training set based on PNI, age, gender, length of stay (LOS) in hospital, platelets (PLT), ethnicity, LOS in ICU, systolic blood pressure (SBP), diastolic blood pressure (DBP), heart rate, glucose, AKI stage, atrial fibrillation (AF), vasopressor, renal replacement therapy (RRT), and mechanical ventilation. The testing set was applied as the internal validation of the model with an AUC of 0.778 (95% CI: 0.754–0.801). In conclusion, PNI accompanied by age, gender, ethnicity, SBP, DBP, heart rate, PLT, glucose, AF, RRT, mechanical ventilation, vasopressor, AKI stage, LOS in ICU, and LOS in hospital exhibited a good predictive value for one-year mortality of AKI patients.

## 1. Introduction

Acute kidney injury (AKI) is a common complication of acute illnesses that is defined as an acute increase in serum creatinine (SCr) and/or a decline in urine volume in the clinic [1]. More than 13 million people suffered from AKI per year all over the world, and nearly 1.7 million deaths were caused by AKI [2]. AKI occurs in about 10%–15% of patients in hospital and over 50% of patients in the intensive care (ICU) patients, which increases the risk of cardiovascular events and progression to chronic kidney disease [3]. Although the supportive care for hospitalized AKI patients has improved the treatments of these patients, the survival is still poor [4]. The mortality rate in AKI patients is as high as 20% and that in the ICUs may reach up to 50% [5]. Predicting the prognosis of patients with AKI is essential for making timely interventions to improve the survival of those patients.

The article "Prediction Models for One-Year Survival of Adult Patients with Acute Kidney Injury: A Longitudinal Study Based on the Data from the Medical Information Mart for Intensive Care III Database" was retracted in 2023. Reasons: suspected computer-generated content; unreliable results or conclusions; lack of ethics approval or compliance; missing or withdrawn patient consent.

At present, multiple pieces of evidence indicated that the prognosis of AKI might be associated with various factors. Sheng et al. found that N-terminal pro-B-type natriuretic peptide was a predictor for the prognosis of AKI patients [6]. Jiao et al. identified that age and lactate levels might be associated with the prognosis of AKI patients [7]. As indicated in previous studies, one of the pathophysiologies of AKI is inflammation [8]. Inflammation-associated indexes including prognostic nutritional index (PNI), platelet-to-lymphocyte ratio (PLR), neutrophil percentage-to-albumin ratio (NPAR), and neutrophil-to-lymphocyte ratio (NLR) were frequently reported to be effective predictors for various diseases. Itoh et al. identified that patients with low PNI were associated with poor clinical outcomes in pancreatic ductal adenocarcinoma patients [9]. NLR and PLR were also identified to be associated with the prognosis of pulmonary embolism patients [10]. In a study by Wang et al., the increased NPAR level on admission was found to be associated with elevated all-cause mortality of patients in cardiac intensive care unit [11]. Additionally, PNI [12], PLR [13], NPAR [14], and NLR [15] were identified to be important prognostic biomarkers for AKI. Several studies reported that factors including age, AKI types, plasma endostatin, central nervous system failure, respiratory failure, hypotension, and acute tubular necrosis-individual severity index score were predictors for the mortality of AKI patients [16, 17]. Prediction models were established based on the predictors [16–18]. A systematic review including 12 prediction models for the survival of AKI patients showed that the predictive values of these models ranged from 0.6 to 0.9 and some of the models had poor predictive performance [19]. In addition, the prediction values of these important inflammation biomarkers including PNI, PLR, NPAR, and NLR were still elusive.

The purpose of our study was to construct prediction models for one-year prognosis in adult AKI patients based on PNI, PLR, NPAR, and NLR, respectively, using the data from Medical Information Mart for Intensive Care III (MIMIC-III). The predictive performance of these four models alone or combined with other predictors was compared to identify a better model for the prediction of one-year survival of adult patients with AKI.

The article "Prediction Models for One-Year Survival of Adult Patients with Acute Kidney Injury: A Longitudinal Study Based on the Data from the Medical Information Mart for Intensive Care III Database" was retracted in 2023. Reasons: suspected computer-generated content; unreliable results or conclusions; lack of ethics approval or compliance; missing or withdrawn patient consent.

## 2. Methods

### 2.1. Study Setting and Population

This was a cohort study including 22745 patients with AKI from MIMIC-III between June 2001 and October 2012. MIMIC-III is a free database including the vital signs, medications, laboratory measurements, observations and notes charted by care providers, fluid balance, procedure codes, diagnostic codes, imaging reports, hospital length of stay, and survival data in patients from critical care units (CCUs) in the Beth Israel Deaconess Medical Center in Boston, Massachusetts [20]. The Institutional Review Boards of Beth Israel Deaconess Medical Center (Boston, MA) and the Massachusetts Institute of Technology (Cambridge, MA) provided approval on the project. AKI patients were diagnosed according to the definition of Kidney Disease: Improving Global Outcomes (KDIGO); that is, the SCr level is increased by 0.3 mg/dl within 48 hours or to 1.5 times the baseline value, which is known or presumed to have occurred within the prior 7 days or a urine volume of <0.5 mL/kg/h for 6 hours [21]. Patients who were aged <18 years, those who died within 24 h of ICU admission, and people who had no data on neutrophil (NEUT), albumin, and lymphocyte (LYM) were excluded. Finally, 6050 patients were involved in our study. The detailed screen process of participants is shown in Figure 1. All the patients were divided into the training set (*n* = 4538) and the testing set (*n* = 1512) at a ratio of 7.5 : 2.5. This study was conducted in accordance with relevant guidelines and regulations. The individual patient consent in our study was not needed as the project did not impact clinical care and all protected health information was deidentified.

### 2.2. Outcome Variables

The outcome variable was to evaluate the death in AKI patients within one year of admission to ICU. The follow-up was one year from the first day of ICU admission. If patients were dead, the follow-up was ended. Those who survived were defined as patients who were alive at the end of the follow-up.

### 2.3. Potential Predictors

The data analyzed were extracted via Structured Query Language (SQL) with MySQL tools (version 5.6.24) including gender, ethnicity (Asian, African American, Hispanic, White, or others), marital status (married, not married, or widowed), age (years), length of stay (LOS) in hospital (day), LOS in ICU (day), first care unit (CCU, the cardiac surgery recovery unit (CSRU), medical intensive care unit (MICU), neonatal intensive care unit (NICU), surgical intensive care unit (SICU), trauma and surgical intensive care unit (TSICU)), AKI stage 48 h (stage 1, stage 2, or stage 3), vasopressor, congestive heart failure, hypertension, chronic obstructive pulmonary disease (COPD), diabetes uncomplicated, renal failure, liver disease, atrial fibrillation (AF), respiratory disease, mechanical ventilation, systolic blood pressure (SBP, mmHg), diastolic blood pressure (DBP, mmHg), heart rate (time/min), respiratory rate (time/min), temperature (°C), peripheral oxygen saturation (SpO_2_, %), mean arterial pressure (MAP, mmHg), prothrombin time (PT, s), white blood cell (WBC, 10^9^/L), LYM (10^9^/L), NEUT (10^9^/L), platelets (PLT, 10^9^/L), hemoglobin (g/uL), red cell distribution width (RDW, %), hematocrit (%), albumin (g/dL), creatinine (mg/dL), international normalized ratio (INR), blood urea nitrogen (BUN, mg/dL), glucose (mg/dL), bicarbonate (mEq/L), sodium (mEq/L), potassium (mEq/L), chloride (mEq/L), calcium (mg/dL), anion gap (mmol/L), total bilirubin (mEq/L), NLR, PLR, NPAR, and PNI. The baseline characteristics were recorded within the first 24 h after patient admission.

The article "Prediction Models for One-Year Survival of Adult Patients with Acute Kidney Injury: A Longitudinal Study Based on the Data from the Medical Information Mart for Intensive Care III Database" was retracted in 2023. Reasons: suspected computer-generated content; unreliable results or conclusions; lack of ethics approval or compliance; missing or withdrawn patient consent.

### 2.4. Definitions of the Variables

NLR=NEUT/LYM, PLR=PLT/LYM, NPAR=NEUT%/albumin, and PNI = 10 × albumin + 0.005 × LYM [22]. AKI stage was defined as follows: stage 1 referred to an increase in SCr to a level ≥1.5 times baseline or 0.3 mg/dl or urine output <0.5 ml/kg/h per 6 h. Stage 2 was defined as an increase in SCr to a level ≥2.0 times baseline or urine output <0.5 mL/kg/h per 12 h. Stage 3 was defined as an increase in SCr to a level ≥3.0 times baseline, an increase in SCr to a level ≥4.0 mg/dl, the initiation of renal replacement therapy (RRT), or urine output <0.5 mL/kg/h per 12 h.

### 2.5. Statistical Analysis

The Shapiro–Wilk test was applied for evaluating the normality of all data. The measurement data with normal distribution were described as mean ± SD, and *t*-test was used for comparison between the two groups. The nonnormal distributed measurement data were displayed as median and quartile spacing M (Q1, Q3), and comparisons between the groups were subjected to the Mann–Whitney U rank-sum test. The enumeration data were expressed as *n* (%). The chi-square test (*χ*^2^) or Fisher's exact probability method were employed for comparing the differences between groups. The outliers or missing values were manipulated, and sensitivity analysis was performed. The least absolute shrinkage and selection operator (LASSO) regression was utilized to screen possible covariates. Three models were constructed. Model 1 was the crude model. Model 2 was adjusted for the democratic characteristics including age, sex, and race, and Model 3 was adjusted for variables with statistical difference screened by LASSO regression including age, gender, ethnicity, SBP, heart rate, PLT, BUN, glucose, AF, RRT, mechanical ventilation, vasopressor, AKI stage, LOS in ICU, and LOS in hospital. Furthermore, the samples were randomly divided into the training set and the testing set at a ratio of 7.5 : 2.5, and the prediction models were constructed in the training set and verified in the testing set by random forest. The prediction values of the models were measured via the sensitivity, specificity, negative prediction value (NPV), positive prediction value (PPV), AUC, and accuracy. Receiver operator characteristic (ROC) curves and variable importance diagram were plotted. Survival outcomes were analyzed through the Kaplan–Meier method and log-rank tests. R (v3.6.3) was applied for data cleaning and preprocessing, and Python 3.7.4 was used for constructing the prediction models. *P* < 0.05 was considered statistically significant.

The article "Prediction Models for One-Year Survival of Adult Patients with Acute Kidney Injury: A Longitudinal Study Based on the Data from the Medical Information Mart for Intensive Care III Database" was retracted in 2023. Reasons: suspected computer-generated content; unreliable results or conclusions; lack of ethics approval or compliance; missing or withdrawn patient consent.

## 3. Results

### 3.1. Sensitivity Analysis after the Manipulation of the Outliers or Missing Values

There were 2 (0.03%) outliers in PLT, 2 (0.03%) outliers in total bilirubin, 1 (0.02%) outlier in creatinine, and 1 (0.02%) outlier in albumin, which were assigned as the maximum value excluding outliers, and then, the missing values were randomly interpolated. Sensitivity analysis was conducted, and the results showed that there was no statistical difference between the data before or after the manipulation of the outliers or missing values (Table 1).

### 3.2. The Baseline Characteristics of Participants

In this study, 22745 patients with AKI from MIMIC-III were included. After excluding patients aged <18 years (*n* = 277), participants died within 24 h of ICU admission (*n* = 572), and subjects without the data on neutrophil, albumin, and lymphocyte (*n* = 15846), 6050 patients were included. In the death group (*n* = 2525), the median age was 73.56 years, the median LOS in hospital was 9.00 days, and the median LOS in ICU was 4.31 days. 933 (36.95%) patients were at AKI stage 3. The median NLR was 10.20, the median PLR was 219.12, the median NPAR was 27.50, and the median PNI was 34.31. Among the survival group (*n* = 3525), the median age was 63.05 years, the median LOS in hospital was 9.38 days, the median LOS in ICU was 3.65 days, and 1027 (29.13%) participants were at AKI stage 1. The median NLR was 8.14, the median PLR was 193.97, the median NPAR was 24.41, and the median PNI was 38.85 (Table 2).

The article "Prediction Models for One-Year Survival of Adult Patients with Acute Kidney Injury: A Longitudinal Study Based on the Data from the Medical Information Mart for Intensive Care III Database" was retracted in 2023. Reasons: suspected computer-generated content; unreliable results or conclusions; lack of ethics approval or compliance; missing or withdrawn patient consent.

### 3.3. Association between NLR, PLR, NPAR, PNI, and One-Year Mortality in AKI Patients

LASSO regression screened out the important covariables including age, SBP, DBP, heart rate, PLT, BUN, and glucose with statistical differences between the death group and the survival group. Three models were established, and the results showed that in model 1, NLR (OR = 1.348, 95% CI: 1.230–1.478), PLR (OR = 1.232, 95% CI: 1.113–1.363), and NPAR (OR = 1.558, 95% CI: 1.350–1.799) were associated with the increased risk of one-year mortality in AKI patients, while PNI (OR = 0.017, 95% CI: 0.010–0.027) was associated with decreased risk of one-year mortality in AKI patients. In model 2, after adjusting for age, gender, and ethnicity, NLR was associated with 1.328-fold risk of one-year mortality in AKI patients (OR = 1.328, 95% CI: 1.210–1.458), PLR was linked with 1.216 times risk of one-year mortality in AKI patients (OR = 1.216, 95% CI: 1.097–1.347), and NPAR was correlated with 1.526-fold risk of one-year mortality in AKI patients (OR = 1.526, 95% CI: 1.319–1.766). NLR decreased the risk of one-year mortality in AKI patients by 0.985 times (OR = 0.015, 95% CI: 0.009–0.025). In model 3, age, gender, ethnicity, SBP, DBP, heart rate, PLT, glucose, AF, RRT, mechanical ventilation, vasopressor, AKI stage, LOS in ICU, and LOS in hospital were adjusted. The results depicted that NLR (OR = 1.261, 95% CI: 1.145–1.388), PLR (OR = 1.295, 95% CI: 1.152–1.445), and NPAR (OR = 1.476, 95% CI: 1.261–1.726) were associated with an increased risk of one-year mortality in AKI patients, while PNI (OR = 0.035, 95% CI: 0.020–0.059) was associated with a decreased risk of one-year mortality in AKI patients (Table 3, Figure 2). Additionally, the logistical models were also constructed in the data with 21896 samples, and the results were similar to the above (Table 4).

### 3.4. Equilibrium Test in the Training Set and the Testing Set

The samples were randomly divided into the training set (*n* = 4538) and the testing set (*n* = 1512), and the equilibrium test was performed in the training set and the testing set. The data in Table 5 revealed that there was no statistical difference between the data in the training set and the testing set.

### 3.5. Establishment of the Random Forest Models

The random forest models for predicting one-year mortality in AKI patients were, respectively, constructed based on PLR, NLR, NPAR, and PNI. The AUCs of PLR, NLR, NPAR, and PNI were 0.592 (95% CI: 0.576–0.609), 0.620 (95% CI: 0.604–0.637), 0.614 (95% CI: 0.597–0.631), and 0.663 (95% CI: 0.647–0.679) in the training set, respectively. In the testing set, the AUCs of PLR, NLR, NPAR, and PNI were 0.552 (95% CI: 0.522–0.581), 0.582 (95% CI: 0.562–0.603), 0.600 (95% CI: 0.571–0.629), and 0.662 (95% CI: 0.634–0.689), respectively (Figure 3).

The article "Prediction Models for One-Year Survival of Adult Patients with Acute Kidney Injury: A Longitudinal Study Based on the Data from the Medical Information Mart for Intensive Care III Database" was retracted in 2023. Reasons: suspected computer-generated content; unreliable results or conclusions; lack of ethics approval or compliance; missing or withdrawn patient consent.

Random forest models were also separately constructed combining PLR, NLR, NPAR, or PNI with the statistical variables involved in the multivariable regression models including age, gender, ethnicity, LOS in hospital, PLT, LOS in ICU, SBP, DBP, heart rate, glucose, AF, AKI stage, vasopressor, RRT, and mechanical ventilation. In the training set of the model based on PLR, NLR, NPAR, and PNI, the sensitivity was 0.969 (95% CI: 0.962–0.975), 0.937 (95% CI: 0.927–0.946), 0.911 (95% CI: 0.901–0.922), and 0.981 (95% CI: 0.976–0.986). The specificity was 0.740 (95% CI: 0.720–0.760), 0.666 (95% CI: 0.644–0.687), 0.815 (95% CI: 0.797–0.833), and 0.781 (95% CI: 0.763–0.800). The PPV was 0.841 (95% CI: 0.828–0.854), 0.799 (95% CI: 0.785–0.813), 0.875 (95% CI: 0.863–0.887), and 0.864 (95% CI: 0.852–0.877). The NPV was 0.944 (95% CI: 0.932–0.955), 0.881 (95% CI: 0.864–0.898), 0.866 (95% CI: 0.850–0.882), and 0.966 (95% CI: 0.957–0.975). The AUC was 0.938 (95% CI: 0.931–0.945), 0.891 (95% CI: 0.882–0.901), 0.936 (95% CI: 0.929–0.944), and 0.964 (95% CI: 0.959–0.969). The accuracy was 0.874 (95% CI: 0.865–0.884), 0.872 (95% CI: 0.862–0.881), 0.825 (95% CI: 0.814–0.836), and 0.898 (95% CI: 0.890–0.907). The sensitivity, specificity, NPV, AUC, and accuracy in the model based on PNI were statistically higher than in the models based on PLR, NLR, and NPAR (*P* < 0.05). The PPV in the model based on PNI was statistically higher than in the models based on PLR and NLR (*P* < 0.05). In the testing set, the sensitivity, PPV, NPV, AUC, and accuracy were 0.834 (95% CI: 0.809–0.859), 0.701 (95% CI: 0.673–0.729), 0.706 (95% CI: 0.666–0.747), 0.758 (95% CI: 0.734–0.783), and 0.703 (95% CI: 0.680–0.726) in the model based on PLR. The sensitivity, AUC, and accuracy were 0.826 (95% CI: 0.801–0.851), 0.759 (95% CI: 0.735–0.783), and 0.709 (95% CI: 0.686–0.732) in the model based on NLR. The sensitivity, PPV, NPV, AUC, and accuracy were 0.849 (95% CI: 0.825–0.873), 0.702 (95% CI: 0.675–0.730), 0.723 (95% CI: 0.683–0.764), 0.768 (95% CI: 0.744–0.792), and 0.698 (95% CI: 0.675–0.721) in the model based on NPAR. The sensitivity, PPV, NPV, AUC, and accuracy were 0.836 (95% CI: 0.812–0.861), 0.708 (95% CI: 0.680–0.735), 0.714 (95% CI: 0.674–0.754), 0.778 (95% CI: 0.754–0.801), and 0.710 (95% CI: 0.687–0.733) in the model based on PNI (Table 6, Figure 4). The model based on PNI, age, gender, ethnicity, AF, LOS in hospital, PLT, LOS in ICU, SBP, DBP, heart rate, glucose, AKI stage, vasopressor, RRT, and mechanical ventilation showed a better predictive value than others and was selected as the final prediction model. The survival curves of actual survival of patients with predicted survival or death outcomes through the prediction model based on PLR, NLR, NPAR, and PNI are, respectively, presented in Supplementary Figures 1–4. The variable importance diagram from the random forest model delineated that age, PNI, and LOS in hospital were the most important variables associated with one-year mortality in AKI patients (Figure 5).

The article "Prediction Models for One-Year Survival of Adult Patients with Acute Kidney Injury: A Longitudinal Study Based on the Data from the Medical Information Mart for Intensive Care III Database" was retracted in 2023. Reasons: suspected computer-generated content; unreliable results or conclusions; lack of ethics approval or compliance; missing or withdrawn patient consent.

## 4. Discussion

In this study, the data of 6050 AKI patients were collected from the MIMIC-III database to, respectively, evaluate the predictive values of PLR, NLR, NPAR, and PNI in the one-year mortality of AKI patients. The results revealed that PLR, NLR, and NPAR were associated with an increased risk of one-year mortality in AKI patients, while PNI was associated with a decreased risk of one-year mortality in AKI patients. The predictive value of random forest model based on PNI was higher than random forest models based on PLR, NLR, or NPAR. After including the variables in the multivariable model into the prediction model, PNI presented a better predictive performance for one-year mortality in AKI patients. The findings of this study might highlight the predictive value of PNI in the prognosis of AKI patients. PNI might help identify patients with high risk of mortality and provide timely interventions to improve the outcomes of these patients.

Systemic inflammation is an integral part of disease progression in critical illness and causes an increased risk of mortality [23]. The inflammatory response plays a vital part in the development and progression of AKI [24]. NLR, a combination of NEUT and LYM counts, serves as a readily available index of systemic inflammation [25]. NLR reflects the balance between innate (NEUT) and adaptive (LYM) immune responses, and NLR elevation was associated with increased concentrations of pro-inflammatory cytokines [26]. Chen et al. found that NLR was a marker for AKI progression and mortality in critically ill people [15]. Fan et al. also indicated that NLR increased the risk of 30-day all-cause mortality in critically ill AKI patients by 0.37 times and the risk of 90-day all-cause mortality by 0.32 times [27]. These findings supported the results in this study, depicting that NLR increased the risk of one-year mortality among AKI patients. PLR is another important inflammation index, and high PLR level was associated with poor prognosis in AKI [13, 28]. This was allied with the results in this study, which showed that PLR was a risk factor for one-year mortality among AKI patients. In the acute inflammatory status, PLT is overactivated and LYM is apoptotic, reflecting the imbalance between PLT and LYM, which might cause immunodeficiency, organ failure, metabolism disorder, and a mismatch between oxygen supply and demand, and ultimately led to death [29, 30]. Serum albumin protects the kidneys from toxic substances and maintains optimal colloid pressure to ensure renal perfusion [31]. Herein, NPAR was also identified to be a risk factor for one-year mortality in patients with AKI. Albumin accounts for more than half of the serum body's composition, which modulates osmotic pressure and exerts antioxidant and anti-inflammatory effects [32, 33]. NPAR is an inflammation biomarker obtained from NEUT percentage-to-albumin ratio, which was established in previous studies to serve as a prognostic biomarker for mortality in AKI patients [14, 34]. PNI, calculated from the serum albumin concentration and LYM, is an index reflecting chronic inflammation, immune system, and nutritional status in patients [35]. Hu et al. demonstrated that each 1 score decrease in PNI resulted in a 2.2% increase in the risk of in-hospital mortality and 1.6% increase in the risk of two-year mortality in AKI patients. This gave support to our findings, depicting that PNI was a protective prognostic factor for AKI patients. This may be because 10%–25% of the body protein content was lost within 10 days after admission in most critically ill patients [36]. Serum albumin is a common indicator of nutritional status, and for AKI patients in ICUs, nutritional interventions should be provided to improve the outcomes in those patients [37]. In this study, the variable importance diagram from random forest model delineated that age, LOS in hospital, and LOS in ICU were the most important variables influencing the outcomes of AKI patients. These were evidenced by previous studies. A former study indicated that older age was associated with increased in-hospital mortality risk in AKI patients who underwent an operation [38]. The LOS in hospital and LOS in ICU were important indicators for evaluating the severity of AKI in patients, and patients with longer LOS in hospital and LOS in ICU were associated with a higher risk of death [39].

The article "Prediction Models for One-Year Survival of Adult Patients with Acute Kidney Injury: A Longitudinal Study Based on the Data from the Medical Information Mart for Intensive Care III Database" was retracted in 2023. Reasons: suspected computer-generated content; unreliable results or conclusions; lack of ethics approval or compliance; missing or withdrawn patient consent.

This study established different prediction models based on PLR, NLR, NPAR, and PNI, respectively. The prediction model established based on PNI showed good predictive value for one-year mortality in AKI patients. Additionally, the prediction model including PNI, age, gender, ethnicity, LOS in hospital, PLT, LOS in ICU, SBP, DBP, heart rate, glucose, AKI stage, AF, vasopressor, RRT, and mechanical ventilation presented a better predictive value with an AUC of 0.964. At present, several prediction models for the mortality of AKI patients were established. A prediction model based on plasma endostatin level combined with sequential organ failure assessment (SOFA) score and AKI classification showed an AUC of 0.833 [11]. Another prediction model constructed according to KDIGO criteria showed an AUC value of 0.832 [12]. Yao et al. constructed a prediction model for in-hospital death of patients with AKI based on age, mechanical ventilation, albumin value, C-reactive protein, surgery, and vasoactive drugs, and the AUC was 0.886 [40]. The AUCs in these studies were lower than the AUC in our study. Li et al. established a prognostic model for critically ill AKI patients and evaluated the AUC (0.716), sensitivity (0.719), specificity (0.601), PPV (0.180), and NPV (0.047) of the model, but the predictive value was poor than the model in our study [18]. Compared with previous prediction models for the mortality in AKI patients, our model had a high AUC value and also high sensitivity, specificity, NPV, PPV, and accuracy. The predictors included in our model were common variables and easy to obtain. Clinicians can quickly predict the outcomes of AKI patients and identify patients at high risk. As early interventions are the keys to successful rescue and low mortality in AKI patients, timely treatments should be provided to those patients with high risk of mortality.

This study had several strengths. Firstly, the outliers and missing values were manipulated and sensitivity analysis was performed, and the results of our study might be more reliable. Limitations also existed in our study. Firstly, most of the patients included in this study were elderly people, so the prediction model might be more suitable for identifying the mortality of middle-aged and elderly people with AKI. Secondly, external validation of the model was not performed. Thirdly, the reasons causing AKI were not included, and the outcomes of AKI patients with different reasons might be different. Fourthly, we only analyzed the associations of baseline PNI, PLR, NPAR, and NLR evaluated during the admission to ICUs with the outcomes of AKI patients, and the effects of PNI, PLR, NPAR, and NLR trajectories and the outcome of AKI patients were not evaluated. In the future, more well-designed prospective studies were required to verify the findings of our study.

## 5. Conclusions

This study evaluated the predictive values of PLR, NLR, NPAR, and PNI in the one-year mortality of AKI patients and established several prediction models for one-year mortality of those patients based on the data of 6050 AKI patients from the MIMIC-III database. The results revealed that PLR, NLR, and NPAR were associated with an increased risk of one-year mortality in AKI patients, while PNI was associated with a decreased risk of one-year mortality in AKI patients. The prediction model of PNI accompanied by age, gender, ethnicity, SBP, heart rate, PLT, BUN, glucose, AF, RRT, mechanical ventilation, vasopressor, AKI stage, LOS in ICU, and LOS in hospital exhibited a good predictive value for one-year mortality of AKI patients. The results might help identify AKI patients with high risk of mortality and provide timely interventions to improve their outcomes.

The article "Prediction Models for One-Year Survival of Adult Patients with Acute Kidney Injury: A Longitudinal Study Based on the Data from the Medical Information Mart for Intensive Care III Database" was retracted in 2023. Reasons: suspected computer-generated content; unreliable results or conclusions; lack of ethics approval or compliance; missing or withdrawn patient consent.

## Figures and Tables

**Figure 1:** Detailed flow chart showing the screen process of participants in this study.

**Figure 2:** Forest plot of results from univariate and multivariate analysis depicting the association between NLR, PLR, NPAR, PNI, and one-year mortality in AKI patients.

**Figure 3:** ROC curves showing the AUCs of prediction model based on PLR, NLR, NPAR, or PNI for one-year mortality of AKI patients in the training set (left panel) and the testing set (right panel).

**Figure 4:** ROC curves showing the AUCs of prediction model based on PLR, NLR, NPAR, or PNI combined with other predictors for one-year mortality of AKI patients in the training set (left panel) and the testing set (right panel).

**Figure 5:** Variable importance diagram revealing the importance of variables influencing the mortality in AKI patients.

**Table 1:** Sensitivity analysis after the manipulation of the outliers or missing values.

Variable	Missing data	After (*n* = 6050)	Before (*n* = 6050)	Statistical magnitude	*P*
Marital status, *n* (%)				*χ* ^2^ = 0.536	0.765
Married	402 (6.64)	2887 (47.72)	2660 (47.10)		
Not married		2166 (35.80)	2036 (36.05)		
Widowed		997 (16.48)	952 (16.86)		
Ethnicity, *n* (%)				*χ* ^2^ = 2.277	0.685
Asian	724 (11.97)	173 (2.86)	143 (2.68)		
African American		605 (10.00)	567 (10.65)		
Hispanic		179 (2.96)	169 (3.17)		
Others		165 (2.73)	152 (2.85)		
White		4928 (81.45)	4295 (80.64)		
Congestive heart failure, *n* (%)				*χ* ^2^ = 0.000	0.984
Yes	9 (1.49)	2025 (33.47)	2023 (33.49)		
No		4025 (66.53)	4018 (66.51)		
Hypertension, *n* (%)				*χ* ^2^ = 0.000	0.999
Yes	7 (1.16)	3377 (55.82)	3373 (55.82)		
No		2673 (44.18)	2670 (44.18)		
COPD, *n* (%)				*χ* ^2^ = 0.001	0.981
Yes	9 (1.49)	1396 (23.07)	1395 (23.09)		
No		4654 (76.93)	4646 (76.91)		
Diabetes uncomplicated, *n* (%)				*χ* ^2^ = 0.000	0.992
Yes	7 (1.16)	1334 (22.05)	1332 (22.04)		
No		4716 (77.95)	4711 (77.96)		
Renal failure, *n* (%)				*χ* ^2^ = 0.001	0.978
Yes	9 (1.49)	1202 (19.87)	1199 (19.85)		
No		4848 (80.13)	4842 (80.15)		
Liver disease, *n* (%)				*χ* ^2^ = 0.000	0.986
Yes	9 (1.49)	1205 (19.92)	1204 (19.93)		
No		4845 (80.08)	4837 (80.07)		
Mechanical ventilation, *n* (%)				*χ* ^2^ = 0.002	0.967
Yes	1 (0.02)	284 (4.69)	283 (4.68)		
No		5766 (95.31)	5766 (95.32)		
SBP, mean ± SD	22 (0.36)	120.22 ± 23.42	120.20 ± 23.45	*t* = 0.05	0.963
DBP, mean ± SD	22 (0.36)	61.22 ± 15.55	61.21 ± 15.57	*t* = 0.02	0.984
Heart rate, mean ± SD	21 (0.35)	86.90 ± 18.70	86.91 ± 18.72	*t* = −0.02	0.982
Respiratory rate, mean ± SD	21 (0.35)	19.78 ± 6.23	19.78 ± 6.24	*t* = 0.00	0.996
Temperature, mean ± SD	25 (0.41)	36.84 ± 0.84	36.84 ± 0.84	*t* = −0.03	0.978
SpO_2_, mean ± SD	22 (0.36)	96.95 ± 3.64	96.95 ± 3.65	*t* = −0.02	0.984
MAP, mean ± SD	21 (0.35)	78.64 ± 16.64	78.63 ± 16.66	*t* = 0.03	0.977
WBC, *M* (*Q*_1_, *Q*_3_)	1 (0.02)	11.50 (7.90, 16.50)	11.50 (7.90, 16.50)	*Z* = −0.009	0.993
PLT, *M* (*Q*_1_, *Q*_3_)	2 (0.03)	213.00 (143.00, 292.00)	213.00 (143.00, 292.00)	*Z* = −0.017	0.987
Hemoglobin, mean ± SD	4 (0.06)	11.25 ± 2.34	11.25 ± 2.34	*t* = 0.03	0.980
RDW, mean ± SD	5 (0.08)	15.46 ± 2.32	15.46 ± 2.32	*t* = 0.02	0.983
Hematocrit, mean ± SD	1 (0.02)	33.61 ± 6.79	33.61 ± 6.79	*t* = 0.01	0.995
Creatinine, *M* (*Q*_1_, *Q*_3_)	1 (0.02)	1.20 (0.80, 2.00)	1.20 (0.80, 2.00)	*Z* = 0.000	1.000
INR, *M* (*Q*_1_, *Q*_3_)	192 (3.17)	1.30 (1.10, 1.70)	1.30 (1.10, 1.70)	*Z* = −0.109	0.913
Glucose, *M* (*Q*_1_, *Q*_3_)	2 (0.03)	134.00 (106.00, 173.00)	134.00 (106.00, 173.00)	*Z* = −0.012	0.991
Bicarbonate, mean ± SD	4 (0.06)	22.73 ± 5.44	22.73 ± 5.44	*t* = −0.07	0.941
Potassium, mean ± SD	4 (0.06)	4.30 ± 0.91	4.30 ± 0.91	*t* = −0.00	0.999
Chloride, mean ± SD	441 (7.29)	104.93 ± 6.84	104.93 ± 6.96	*t* = 0.02	0.981
Calcium, mean ± SD	155 (2.56)	8.24 ± 1.05	8.24 ± 1.05	*t* = −0.06	0.952
Anion_gap, mean ± SD	2 (0.03)	16.10 ± 4.88	16.10 ± 4.88	*t* = 0.00	0.999
Bilirubin 3, *M* (*Q*_1_, *Q*_3_)	857 (14.17)	0.70 (0.40, 1.40)	0.70 (0.40, 1.50)	*Z* = −0.956	0.339

LOS: length of stay, CSRU: cardiac surgery recovery unit, MICU: medical intensive care unit, NICU: neonatal intensive care unit, SICU: surgical intensive care unit, TSICU: trauma and surgical intensive care unit, AKI: acute kidney injury, COPD: chronic obstructive pulmonary disease, AF: atrial fibrillation, SBP: systolic blood pressure, DBP: diastolic blood pressure, SpO_2_: peripheral oxygen saturation, MAP: mean arterial pressure, PT: prothrombin time, WBC: white blood cell, LYM: lymphocyte, NEUT: neutrophil, PLT: platelets, RDW: red cell distribution width, INR: international normalized ratio.

The article "Prediction Models for One-Year Survival of Adult Patients with Acute Kidney Injury: A Longitudinal Study Based on the Data from the Medical Information Mart for Intensive Care III Database" was retracted in 2023. Reasons: suspected computer-generated content; unreliable results or conclusions; lack of ethics approval or compliance; missing or withdrawn patient consent.

**Table 2:** Comparisons of characteristics in participants who survived or dead with AKI.

Variable	Total (*n* = 6050)	Death group (*n* = 2525)	Survival group (*n* = 3525)	Statistical magnitude	*P*
Gender (female), *n* (%)	3333 (55.09)	1420 (56.24)	1913 (54.27)	*χ* ^2^ = 2.303	0.129
Ethnicity, *n* (%)				*χ* ^2^ = 21.807	<0.001
Asian	173 (2.86)	97 (3.84)	76 (2.16)		
African American	605 (10.00)	226 (8.95)	379 (10.75)		
Hispanic	179 (2.96)	67 (2.65)	112 (3.18)		
Others	165 (2.73)	63 (2.50)	102 (2.89)		
White	4928 (81.45)	2072 (82.06)	2856 (81.02)		
Marital status, *n* (%)				*χ* ^2^ = 68.946	<0.001
Married	2887 (47.72)	1249 (49.47)	1638 (46.47)		
Not married	2166 (35.80)	771 (30.53)	1395 (39.57)		
Widowed	997 (16.48)	505 (20.00)	492 (13.96)		
Age, *M* (*Q*_1_, *Q*_3_)	67.52 (54.33, 79.56)	73.56 (60.64, 82.75)	63.05 (51.24, 75.87)	*Z* = 19.022	<0.001
LOS in hospital, *M* (*Q*_1_, *Q*_3_)	9.19 (5.47, 16.66)	9.00 (5.10, 16.77)	9.38 (5.68, 16.63)	*Z* = −1.741	0.082
LOS in ICU, *M* (*Q*_1_, *Q*_3_)	3.91 (2.14, 8.07)	4.31 (2.38, 8.76)	3.65 (2.02, 7.67)	*Z* = 6.480	<0.001
First care unit, *n* (%)				*χ* ^2^ = 2.285	0.809
CCU	812 (13.42)	331 (13.11)	481 (13.65)		
CSRU	1597 (26.40)	670 (26.53)	927 (26.30)		
MICU	2010 (33.22)	836 (33.11)	1174 (33.30)		
NICU	61 (1.01)	30 (1.19)	31 (0.88)		
SICU	883 (14.60)	377 (14.93)	506 (14.35)		
TSICU	687 (11.36)	281 (11.13)	406 (11.52)		
AKI stage 48 hr, *n* (%)				*χ* ^2^ = 226.572	<0.001
1	1538 (25.42)	511 (20.24)	1027 (29.13)		
2	2880 (47.60)	1081 (42.81)	1799 (51.04)		
3	1632 (26.98)	933 (36.95)	699 (19.83)		
Vasopressor (yes), *n* (%)	1264 (20.89)	623 (24.67)	641 (18.18)	*χ* ^2^ = 37.480	<0.001
Congestive heart failure (yes), *n* (%)	2025 (33.47)	990 (39.21)	1035 (29.36)	*χ* ^2^ = 64.051	<0.001
Hypertension (yes), *n* (%)	3377 (55.82)	1362 (53.94)	2015 (57.16)	*χ* ^2^ = 6.195	0.013
CPD (yes), *n* (%)	1396 (23.07)	616 (24.40)	780 (22.13)	*χ* ^2^ = 4.265	0.039
Diabetes uncomplicated (yes), *n* (%)	1334 (22.05)	544 (21.54)	790 (22.41)	*χ* ^2^ = 0.643	0.423
Renal failure (yes), *n* (%)	1202 (19.87)	611 (24.20)	591 (16.77)	*χ* ^2^ = 51.042	<0.001
Liver disease (yes), *n* (%)	1205 (19.92)	619 (24.51)	586 (16.62)	*χ* ^2^ = 57.429	<0.001
AF (yes), *n* (%)	1784 (29.49)	940 (37.23)	844 (23.94)	*χ* ^2^ = 124.867	<0.001
Respiratory disease (yes), *n* (%)	1456 (24.07)	704 (27.88)	752 (21.33)	*χ* ^2^ = 34.516	<0.001
Mechanical ventilation (yes), *n* (%)	5766 (95.31)	2367 (93.74)	3399 (96.43)	*χ* ^2^ = 23.671	<0.001
SBP, mean ± SD	120.22 ± 23.42	116.52 ± 23.43	122.87 ± 23.06	*t* = −10.49	<0.001
DBP (mmHg), mean ± SD	61.22 ± 15.55	58.44 ± 14.84	63.21 ± 15.75	*t* = −12.01	<0.001
Heart rate, mean ± SD	86.90 ± 18.70	88.41 ± 19.31	85.83 ± 18.17	*t* = 5.27	<0.001
Respiratory rate, mean ± SD	19.78 ± 6.23	20.23 ± 6.35	19.46 ± 6.13	*t* = 4.77	<0.001
Temperature, mean ± SD	36.84 ± 0.84	36.74 ± 0.90	36.92 ± 0.79	*t* = −8.16	<0.001
SpO_2_%, mean ± SD	96.95 ± 3.64	96.77 ± 4.33	97.07 ± 3.05	*t* = −3.02	0.003
MAP, mean ± SD	78.64 ± 16.64	76.02 ± 16.16	80.51 ± 16.73	*t* = −10.44	<0.001
PT, *M* (*Q*_1_, *Q*_3_)	13.70 (13.70, 14.90)	13.70 (13.70, 15.80)	13.70 (13.70, 14.50)	*Z* = 9.140	<0.001
WBC, *M* (*Q*_1_, *Q*_3_)	11.50 (7.90, 16.50)	12.30 (8.10, 17.80)	11.20 (7.80, 15.80)	*Z* = 5.107	<0.001
LYM, *M* (*Q*_1_, *Q*_3_)	9.00 (5.20, 15.50)	8.00 (4.30, 13.80)	10.00 (6.00, 16.50)	*Z* = −10.849	<0.001
NEUT, mean ± SD	78.25 ± 15.40	78.20 ± 17.40	78.29 ± 13.80	*t* = −0.21	0.831
PLT, *M* (*Q*_1_, *Q*_3_)	213.00 (143.00, 292.00)	202.00 (122.00, 290.00)	219.00 (156.00, 294.00)	*Z* = −6.454	<0.001
Hemoglobin, mean ± SD	11.25 ± 2.34	10.76 ± 2.26	11.61 ± 2.34	*t* = −14.10	<0.001
RDW, mean ± SD	15.46 ± 2.32	16.25 ± 2.51	14.89 ± 2.00	*t* = 22.68	<0.001
Hematocrit, mean ± SD	33.61 ± 6.79	32.45 ± 6.66	34.45 ± 6.76	*t* = −11.44	<0.001
Albumin, mean ± SD	3.11 ± 0.72	2.91 ± 0.69	3.25 ± 0.70	*t* = −18.55	<0.001
Creatinine, *M* (*Q*_1_, *Q*_3_)	1.20 (0.80, 2.00)	1.40 (0.90, 2.40)	1.10 (0.80, 1.70)	*Z* = 11.533	<0.001
INR, *M* (*Q*_1_, *Q*_3_)	1.30 (1.10, 1.70)	1.40 (1.20, 1.90)	1.28 (1.10, 1.50)	*Z* = 16.021	<0.001
BUN, *M* (*Q*_1_, *Q*_3_)	25.00 (16.00, 43.00)	32.00 (20.00, 52.00)	22.00 (14.00, 35.00)	*Z* = 19.745	<0.001
Glucose, *M* (*Q*_1_, *Q*_3_)	134.00 (106.00, 173.00)	131.00 (104.00, 171.00)	135.00 (108.00, 175.00)	*Z* = −3.217	0.001
Bicarbonate, mean ± SD	22.73 ± 5.44	22.32 ± 5.79	23.02 ± 5.16	*t* = −4.80	<0.001
Sodium, mean ± SD	138.31 ± 5.80	138.10 ± 6.29	138.46 ± 5.42	*t* = −2.29	0.022
Potassium, mean ± SD	4.30 ± 0.91	4.39 ± 0.95	4.24 ± 0.87	*t* = 6.26	<0.001
Chloride, mean ± SD	104.93 ± 6.84	104.81 ± 7.33	105.01 ± 6.46	*t* = −1.13	0.259
Calcium, mean ± SD	8.24 ± 1.05	8.17 ± 1.01	8.29 ± 1.06	*t* = −4.57	<0.001
Anion gap, mean ± SD	16.10 ± 4.88	16.53 ± 4.88	15.79 ± 4.85	*t* = 5.89	<0.001
Bilirubin, *M* (*Q*_1_, *Q*_3_)	0.70 (0.40, 1.40)	0.80 (0.50, 2.00)	0.68 (0.40, 1.20)	*Z* = 9.070	<0.001
NLR, *M* (*Q*_1_, *Q*_3_)	8.94 (4.79, 16.20)	10.20 (5.33, 19.50)	8.14 (4.48, 14.38)	*Z* = 9.372	<0.001
PLR, *M* (*Q*_1_, *Q*_3_)	203.04 (117.50, 353.48)	219.12 (119.67, 398.35)	193.97 (116.42, 323.27)	*Z* = 4.531	<0.001
NPAR, *M* (*Q*_1_, *Q*_3_)	25.70 (21.22, 31.11)	27.50 (22.82, 33.78)	24.41 (20.43, 29.17)	*Z* = 15.374	<0.001
PNI, *M* (*Q*_1_, *Q*_3_)	36.95 (30.93, 43.14)	34.31 (28.62, 40.10)	38.85 (32.88, 44.93)	*Z* = −18.714	<0.001

LOS: length of stay, CSRU: cardiac surgery recovery unit, MICU: medical intensive care unit, NICU: neonatal intensive care unit, SICU: surgical intensive care unit, TSICU: trauma and surgical intensive care unit, COPD: chronic obstructive pulmonary disease, AF: atrial fibrillation, AKI: acute kidney injury, SBP: systolic blood pressure, DBP: diastolic blood pressure, SpO_2_: peripheral oxygen saturation, MAP: mean arterial pressure, PT: prothrombin time, WBC: white blood cell, LYM: lymphocyte, NEUT: neutrophil, PLT: platelets, RDW: red cell distribution width, INR: international normalized ratio, PNI: prognostic nutritional index, PLR: platelet-to-lymphocyte ratio, NPAR: neutrophil percentage-to-albumin ratio, NLR: neutrophil-to-lymphocyte ratio.

The article "Prediction Models for One-Year Survival of Adult Patients with Acute Kidney Injury: A Longitudinal Study Based on the Data from the Medical Information Mart for Intensive Care III Database" was retracted in 2023. Reasons: suspected computer-generated content; unreliable results or conclusions; lack of ethics approval or compliance; missing or withdrawn patient consent.

**Table 3:** Association between NLR, PLR, NPAR, PNI, and one-year mortality in AKI patients.

Variable	Model 1		Model 2		Model 3	
	OR (95% CI)	*P*	OR (95% CI)	*P*	OR (95% CI)	*P*
NLR	1.348 (1.230–1.478)	<0.001	1.328 (1.210–1.458)	<0.001	1.261 (1.145–1.388)	<0.001
PLR	1.232 (1.113–1.363)	<0.001	1.216 (1.097–1.347)	<0.001	1.295 (1.152–1.445)	<0.001
NPAR	1.558 (1.350–1.799)	<0.001	1.526 (1.319–1.766)	<0.001	1.476 (1.261–1.726)	<0.001
PNI	0.017 (0.010–0.027)	<0.001	0.015 (0.009–0.025)	<0.001	0.035 (0.020–0.059)	<0.001

AKI: acute kidney injury, PNI: prognostic nutritional index, PLR: platelet-to-lymphocyte ratio, NPAR: neutrophil percentage-to-albumin ratio, NLR: neutrophil-to-lymphocyte ratio.

**Table 4:** Association between NLR, PLR, NPAR, PNI, and one-year mortality in AKI patients based on the initial data with 21896 AKI patients.

Variable	Model 1		Model 2		Model 3	
	OR (95% CI)	*P*	OR (95% CI)	*P*	OR (95% CI)	*P*
NLR	1.402 (1.293–1.520)	<0.001	1.384 (1.275–1.503)	<0.001	1.255 (1.153–1.365)	<0.001
PLR	1.335 (1.221–1.460)	<0.001	1.324 (1.209–1.450)	<0.001	1.323 (1.197–1.463)	<0.001
NPAR	4.251 (2.926–6.176)	<0.001	4.373 (2.992–6.391)	<0.001	2.915 (1.997–4.256)	<0.001
PNI	0.020 (0.012–0.034)	<0.001	0.018 (0.010–0.030)	<0.001	0.040 (0.023–0.071)	<0.001

AKI: acute kidney injury, PNI: prognostic nutritional index, PLR: platelet-to-lymphocyte ratio, NPAR: neutrophil percentage-to-albumin ratio, NLR: neutrophil-to-lymphocyte ratio.

**Table 5:** Equilibrium test in the training set and the testing set.

Variable	Total (*n* = 6050)	Training (*n* = 4538)	Testing (*n* = 1512)	Statistical magnitude	*P*
LOS in ICU, *M* (*Q*_1_, *Q*_3_)	3.91 (2.14, 8.07)	3.92 (2.11, 8.12)	3.87 (2.20, 7.81)	*Z* = −0.088	0.930
First care unit, *n* (%)				*χ* ^2^ = 8.111	0.150
CCU	812 (13.42)	611 (13.46)	201 (13.29)		
CSRU	1597 (26.40)	1169 (25.76)	428 (28.31)		
MICU	2010 (33.22)	1503 (33.12)	507 (33.53)		
NICU	61 (1.01)	49 (1.08)	12 (0.79)		
SICU	883 (14.60)	689 (15.18)	194 (12.83)		
TSICU	687 (11.36)	517 (11.39)	170 (11.24)		
AKI stage 48 hr, *n* (%)				*χ* ^2^ = 0.240	0.887
1	1538 (25.42)	1160 (25.56)	378 (25.00)		
2	2880 (47.60)	2153 (47.44)	727 (48.08)		
3	1632 (26.98)	1225 (26.99)	407 (26.92)		
Marital status, *n* (%)				*χ* ^2^ = 1.077	0.584
Married	2887 (47.72)	2164 (47.69)	723 (47.82)		
Not married	2166 (35.80)	1614 (35.57)	552 (36.51)		
Widowed	997 (16.48)	760 (16.75)	237 (15.67)		
Ethnicity, *n* (%)				*χ* ^2^ = 1.682	0.794
Asian	173 (2.86)	129 (2.84)	44 (2.91)		
African American	605 (10.00)	444 (9.78)	161 (10.65)		
Hispanic	179 (2.96)	137 (3.02)	42 (2.78)		
Others	165 (2.73)	128 (2.82)	37 (2.45)		
White	4928 (81.45)	3700 (81.53)	1228 (81.22)		
Gender, *n* (%)				*χ* ^2^ = 0.014	0.906
Male	2717 (44.91)	2036 (44.87)	681 (45.04)		
Female	3333 (55.09)	2502 (55.13)	831 (54.96)		
LOS in hospital, *M* (*Q*_1_, *Q*_3_)	9.19 (5.47, 16.66)	9.36 (5.56, 16.75)	8.86 (5.34, 16.18)	*Z* = −1.345	0.179
Age, *M* (*Q*_1_, *Q*_3_)	67.52 (54.33, 79.56)	67.46 (54.02, 79.62)	67.77 (55.23, 79.44)	*Z* = 0.624	0.532
Vasopressor (yes), *n* (%)	1264 (20.89)	947 (20.87)	317 (20.97)	*χ* ^2^ = 0.007	0.936
Congestive heart failure (yes), *n*(%)	2025 (33.47)	1512 (33.32)	513 (33.93)	*χ* ^2^ = 0.189	0.663
Hypertension (yes), *n* (%)	3377 (55.82)	2537 (55.91)	840 (55.56)	*χ* ^2^ = 0.056	0.812
CPD (yes), *n* (%)	1396 (23.07)	1044 (23.01)	352 (23.28)	*χ* ^2^ = 0.048	0.826
Diabetes uncomplicated (yes), *n* (%)	1334 (22.05)	980 (21.60)	354 (23.41)	*χ* ^2^ = 2.179	0.140
Renal failure (yes), *n* (%)	1202 (19.87)	912 (20.10)	290 (19.18)	*χ* ^2^ = 0.599	0.439
Liver disease (yes), *n* (%)	1205 (19.92)	914 (20.14)	291 (19.25)	*χ* ^2^ = 0.570	0.450
AF (yes), *n* (%)	1784 (29.49)	1335 (29.42)	449 (29.70)	*χ* ^2^ = 0.042	0.838
Respiratory disease (yes), *n* (%)	1456 (24.07)	1090 (24.02)	366 (24.21)	*χ* ^2^ = 0.022	0.883
Mechanical ventilation (yes), *n* (%)	5766 (95.31)	4324 (95.28)	1442 (95.37)	*χ* ^2^ = 0.019	0.891
SBP, mean ± SD	120.22 ± 23.42	120.11 ± 23.36	120.55 ± 23.60	*t* = 0.63	0.528
DBP, mean ± SD	61.22 ± 15.55	61.22 ± 15.64	61.22 ± 15.28	*t* = 0.01	0.989
Heart_rate, mean ± SD	86.90 ± 18.70	86.86 ± 18.58	87.03 ± 19.04	*t* = 0.29	0.769
Respiratory_rate, mean ± SD	19.78 ± 6.23	19.78 ± 6.34	19.78 ± 5.92	*t* = 0.00	0.997
Temperature, mean ± SD	36.84 ± 0.84	36.85 ± 0.84	36.83 ± 0.85	*t* = −0.70	0.486
SpO_2_, mean ± SD	96.95 ± 3.64	96.91 ± 3.85	97.08 ± 2.92	*t* = 1.80	0.072
MAP, mean ± SD	78.64 ± 16.64	78.75 ± 16.91	78.29 ± 15.81	*t* = −0.98	0.329
WBC, *M* (*Q*_1_, *Q*_3_)	11.50 (7.90, 16.50)	11.60 (7.90, 16.40)	11.40 (7.70, 16.60)	*Z* = −1.161	0.246
PCT, *M* (*Q*_1_, *Q*_3_)	213.00 (143.00, 292.00)	214.00 (145.00, 293.00)	210.00 (139.00, 291.00)	*Z* = −0.988	0.323
Hemoglobin, mean ± SD	11.25 ± 2.34	11.27 ± 2.31	11.21 ± 2.43	*t* = −0.74	0.457
RDW, mean ± SD	15.46 ± 2.32	15.43 ± 2.27	15.55 ± 2.48	*t* = 1.61	0.107
Hematocrit, mean ± SD	33.61 ± 6.79	33.65 ± 6.69	33.50 ± 7.07	*t* = −0.72	0.474
Albumin, mean ± SD	3.11 ± 0.72	3.11 ± 0.72	3.10 ± 0.73	*t* = −0.17	0.862
Creatinine, *M* (*Q*_1_, *Q*_3_)	1.20 (0.80, 2.00)	1.20 (0.80, 2.00)	1.20 (0.80, 2.00)	*Z* = −0.229	0.819
INR, *M* (*Q*_1_, *Q*_3_)	1.30 (1.10, 1.70)	1.30 (1.10, 1.70)	1.30 (1.10, 1.60)	*Z* = −0.632	0.527
BUN, *M* (*Q*_1_, *Q*_3_)	25.00 (16.00, 43.00)	25.00 (16.00, 42.00)	26.00 (17.00, 44.00)	*Z* = 1.387	0.165
Glucose, *M* (*Q*_1_, *Q*_3_)	134.00 (106.00, 173.00)	134.00 (107.00, 173.00)	133.00 (104.00, 175.00)	*Z* = −1.080	0.280
Bicarbonate, mean ± SD	22.73 ± 5.44	22.75 ± 5.44	22.64 ± 5.45	*t* = −0.67	0.500
Sodium, mean ± SD	138.31 ± 5.80	138.28 ± 5.72	138.40 ± 6.05	*t* = 0.70	0.483
Potassium, mean ± SD	4.30 ± 0.91	4.31 ± 0.92	4.28 ± 0.88	*t* = −1.00	0.315
Chloride, mean ± SD	104.93 ± 6.84	104.96 ± 6.89	104.82 ± 6.68	*t* = −0.71	0.478
Calcium, mean ± SD	8.24 ± 1.05	8.24 ± 1.05	8.22 ± 1.03	*t* = −0.70	0.481
Anion_gap, mean ± SD	16.10 ± 4.88	16.07 ± 4.88	16.17 ± 4.87	*t* = 0.67	0.501
Bilirubin, *M* (*Q*_1_, *Q*_3_)	0.70 (0.40, 1.40)	0.70 (0.40, 1.40)	0.70 (0.40, 1.40)	*Z* = 0.180	0.857
NLR, *M* (*Q*_1_, *Q*_3_)	0.95 (0.68, 1.21)	0.95 (0.68, 1.21)	0.95 (0.69, 1.21)	*Z* = −0.260	0.795
PLR, mean ± SD	2.34 ± 0.51	2.34 ± 0.52	2.32 ± 0.47	*t* = −1.33	0.182
NAR, *M* (*Q*_1_, *Q*_3_)	0.47 (0.26, 0.67)	0.47 (0.27, 0.67)	0.45 (0.26, 0.66)	*Z* = −1.132	0.258
NPAR, *M* (*Q*_1_, *Q*_3_)	0.47 (0.26, 0.67)	0.47 (0.27, 0.67)	0.46 (0.26, 0.66)	*Z* = −1.136	0.256
PNI, mean ± SD	1.56 ± 0.12	1.56 ± 0.12	1.56 ± 0.12	*t* = −0.03	0.979
PT, *M* (*Q*_1_, *Q*_3_)	13.70 (13.70, 14.90)	13.70 (13.70, 14.90)	13.70 (13.70, 14.90)	*Z* = −1.029	0.303

LOS: length of Stay, CSRU: cardiac surgery recovery unit, MICU: medical intensive care unit, NICU: neonatal intensive care unit, SICU: surgical intensive care unit, TSICU: trauma and surgical intensive care unit, COPD: chronic obstructive pulmonary disease, AF: atrial fibrillation, AKI: acute kidney injury, SBP: systolic blood pressure, DBP: diastolic blood pressure, SpO_2_: peripheral oxygen saturation, MAP: mean arterial pressure, PT: prothrombin time, WBC: white blood cell, LYM: lymphocyte, NEUT: neutrophil, PLT: platelets, RDW: red cell distribution width, INR: international normalized ratio, PNI: prognostic nutritional index, PLR: platelet-to-lymphocyte ratio, NPAR: neutrophil percentage-to-albumin ratio, NLR: neutrophil-to-lymphocyte ratio.

The article "Prediction Models for One-Year Survival of Adult Patients with Acute Kidney Injury: A Longitudinal Study Based on the Data from the Medical Information Mart for Intensive Care III Database" was retracted in 2023. Reasons: suspected computer-generated content; unreliable results or conclusions; lack of ethics approval or compliance; missing or withdrawn patient consent.

**Table 6:** Establishment of the random forest models.

Character	Model	Training set	Testing set
Sensitivity (95% CI)	PLR	0.969 (0.962–0.975)^a^	0.834 (0.809–0.859)
	NLR	0.937 (0.927–0.946)^a^	0.826 (0.801–0.851)
	NPAR	0.911 (0.901–0.922)^a^	0.849 (0.825–0.873)
	PNI	0.981 (0.976–0.986)	0.836 (0.812–0.861)

Specificity (95% CI)	PLR	0.740 (0.720–0.760)^a^	0.529 (0.491–0.568)
	NLR	0.666 (0.644–0.687)^a^	0.528 (0.489–0.566)
	NPAR	0.815 (0.797–0.833)^a^	0.523 (0.485–0.561)
	PNI	0.781 (0.763–0.800)	0.542 (0.503–0.580)

PPV (95% CI)	PLR	0.841 (0.828–0.854)^a^	0.701 (0.673–0.729)
	NLR	0.799 (0.785–0.813)^a^	0.699 (0.671–0.727)
	NPAR	0.875 (0.863–0.887)	0.702 (0.675–0.730)
	PNI	0.864 (0.852–0.877)	0.708 (0.680–0.735)

NPV (95% CI)	PLR	0.944 (0.932–0.955)^a^	0.706 (0.666–0.747)
	NLR	0.881 (0.864–0.898)^a^	0.696 (0.655–0.736)
	NPAR	0.866 (0.850–0.882)^a^	0.723 (0.683–0.764)
	PNI	0.966 (0.957–0.975)	0.714 (0.674–0.754)

AUC (95% CI)	PLR	0.938 (0.931–0.945)^a^	0.758 (0.734–0.783)
	NLR	0.891 (0.882–0.901)^a^	0.759 (0.735–0.783)
	NPAR	0.936 (0.929–0.944)^a^	0.768 (0.744–0.792)
	PNI	0.964 (0.959–0.969)	0.778 (0.754–0.801)

Accuracy (95% CI)	PLR	0.874 (0.865–0.884)^a^	0.703 (0.680–0.726)
	NLR	0.872 (0.862–0.881)^a^	0.709 (0.686–0.732)
	NPAR	0.825 (0.814–0.836)^a^	0.698 (0.675–0.721)
	PNI	0.898 (0.890–0.907)	0.710 (0.687–0.733)

a: when compared with PNI, *P* < 0.05, NPV: negative prediction value, PPV: positive prediction value, AUC: area under the curve.

## Data Availability

The datasets generated and/or analyzed during this study are available in the MIMIC repository, https://mimic.mit.edu/.

## Supplementary Materials

Supplementary Materials Supplementary Figure 1. Survival curves of actual survival of patients with predicted survival or death outcomes through the prediction model based on PLR. Supplementary Figure 2. Survival curves of actual survival of patients with predicted survival or death outcomes through the prediction model based on NLR. Supplementary Figure 3. Survival curves of actual survival of patients with predicted survival or death outcomes through the prediction model based on NPAR. Supplementary Figure 4. Survival curves of actual survival of patients with predicted survival or death outcomes through the prediction model based on PNI.
